The article "A Study on Insulation Monitoring Technology of High-Voltage Cables in Underground Coal Mines Based on Decision Tree" was retracted in 2023. Reasons: signs of a paper mill; suspected computer-generated content; unreliable results or conclusions; concerns about the data.

# A Study on Insulation Monitoring Technology of High-Voltage Cables in Underground Coal Mines Based on Decision Tree

**DOI:** 10.1155/2022/2247017

**Published:** 2022-05-23

**Authors:** Wenjun Fu, Ying Xu, Yan Gao

**Affiliations:** ^1^Beijing China Coal Mine Engineering Co., Ltd, Beijing 100013, China; ^2^Liaoning Technical University, Fuxin 123000, China; ^3^China University of Mining and Technology, Beijing 100013, China

## Abstract

The insulation state of high-voltage cables in coal mines directly influences the reliability of power supply in coal mines and the level of safe production. In this paper, the degradation mechanism of cable insulation is analyzed, and an online monitoring technology of cable insulation in coal mines based on decision tree is proposed, the technical principle of the judgment method of cable degradation based on decision tree is studied, the feasibility of this technology is verified through simulation, the existing online monitoring solutions for cable insulation are analyzed, and a wide-area synchronous measurement and monitoring system for cable insulation is designed. This technology has been applied in Chinese coal mine enterprises in China and achieved a good effect.

## 1. Introduction

High-voltage cables are a kind of key equipment for high-voltage, large-capacity, and long-distance power transmission [1]. In 6 kV or 10 kV power supply systems of coal mines in China, power cables are the main power transmission lines, with a coverage rate of above 90% in the power supply lines of coal mines [2, 3]. High-voltage cables are widely used in underground coal mines. The failure of the power cable, which is an important energy transmission element in the power supply system of coal mines, is largely due to the aging of cable insulation [4]. If the insulation state of high-voltage cables in underground coal mines cannot be monitored in real time, it will easily cause the unbalanced operation of the system and affect the reliability of power supply in coal mines and the level of safe production. If the insulation degradation of cables cannot be discovered and measures are not taken in time, it may incur the following hazards:

### 1.1. Asymmetric Operating Voltage of the System

Three-phase symmetry refers to the state of the three-phase three-wire power supply system with same-frequency equal-magnitude voltage and current of each phase with the mutual phase difference of 120 degrees. When cable insulation degrades to a certain degree, the distributed capacitance of the cable will increase, and the insulation resistance will decrease. The asymmetry of three-phase insulation parameters of cables will result in the asymmetry of operating voltage of the system. For electric generators and transformers, in case of the imbalance of three-phase load, if controlling the maximum phase current as the rated value, the remaining two phases cannot be fully loaded, thus reducing the equipment utilization. On the contrary, in order to maintain the rated capacity, it will result in large first-phase overload and magnetic circuit imbalance, causing waveform distortion and increasing the additional losses of the equipment. Long-term asymmetric operating voltage can shorten the service life of other electrical appliances in the system. Meanwhile, the normal service life of cables will also be shortened, which further accelerates the insulation degradation of corresponding cables and forms a vicious circle.

### 1.2. Triggering a Leakage Fault

Among a lot of cable insulating medium defects, the most common is the partial discharge caused by air gaps. Because the dielectric constant of the gas is always less than the dielectric constant of the liquid or solid, and the cable is influenced by process levels and working environments during production, transportation, and use, there may exist air gaps in the insulating layer. Under AC operating voltage, the increase in air gap is increased to produce free electrons and ions are generated in the air gap due to the increase of the surrounding field intensity. The strong ionization reaction between these free electrons and ions in air gap leads to the distortion of the local electric field and decomposes the insulating materials of the air gap wall, followed by a large amount of thermal energy. The high temperature causes carbonization in the air gap, chemical corrosion, and other effects, resulting in the destruction and decomposition of insulating materials near the ionization zone, which also gradually develop deep along the electric field. With the increase in the number of partial discharges, the insulation level may drop continuously or even suffer complete breakdown and trigger a leakage fault. If a leakage fault is not handled properly, it may develop into a grounding or short circuit fault and conduce to override trip and large-scale power failure [5].

### 1.3. Endangering the Safe Operation of Coal Mines

Among all coal mines in China, highly gassy mines account for a vast majority. When underground ventilation is poor, toxin and gas, coal dust, and other flammable substances tend to gather. When the insulation degradation of cables evolves into a breakdown, electric leakage or electric arc is likely to occur. If the energy of electric sparks reaches the minimum ignition point of gas or coal dust, that is, 0.28 mJ, gas explosion will happen and endanger the production of coal mine and the life of workers [6]. If the leakage current is greater than 50 mA, it may cause the premature explosion of electric detonator.

In recent years, underground cable fire accidents have become more and more frequent and serious, which not only influences the normal mining of underground coal resources, but also seriously threatens people's life and property. According to incomplete statistics of accident surveys in China, more than 10 accidents were triggered by cables in coal mining within 7 years from the end of 2007 to 2014, which resulted in more than 100 casualties [7]. The complicated and changeable underground environment and low temperature, humidity, dust, noise, excessively high concentration of gas, and difficulty in monitoring are important factors leading to cable accidents [8]. The air humidity in coal mines is generally above 90%, and there are often drips and drenches. The chambers and roadways have poor heat dissipation conditions and high temperature [9, 10]. The harsh environment of high-voltage cables in underground coal mines will accelerate the aging of cables and facilitate the decline of insulation, which is prone to leakage faults and even intermittent arcs. On the other hand, the nonselective misoperation of single-phase grounding fault will also result in large-scale power failure and have a direct bearing on safe production. Power failure will trigger blowing out and possibly safety accidents, such as accumulation of underground gas and breathing difficulty of workers. In underground where gases and coal dust gather, it is very easy for the electric sparks generated at the time of breakdown of cable insulation to cause explosion accidents and mine casualties. It is a relatively slow process from cable insulation damage to single-phase leakage fault, and the electrical parameters change slowly, so it is imperative to monitor insulation in real time to prevent the occurrence of leakage accidents. Thus, in order to ensure the reliability of power supply and safety production in coal mines, it is essential to monitor and diagnose the insulation state of power cables in real time, so as to improve the safety of high-voltage power supply system in coal mines [11].

In this paper, taking high-voltage cable in underground mine as the research object, the author analyzed the insulation deterioration mechanism, proposed the coal mine cable insulation online monitoring technology based on decision-making tree, estimated the insulation deterioration phase of the cable according to the phase relationship between zero-sequence current and three-phase grounding voltage, redetermined the insulation conductance and distribution capacitance value of the cable using the corresponding calculation formula, and realized accurate judgment of the cable insulation deterioration phase and the degree deterioration. On this basis, a cable insulation monitoring method based on wide-area synchronous measurements is investigated and designed, which is conductive to enhancing the decision-making accuracy.

## 2. Degradation Factors of Cable Insulation

When the cable insulation degrades, the leakage current is tiny and the signal characteristics are not obvious, making it difficult to diagnose the insulation state accurately. The development process of cable insulation is that the insulation is sound when the cables leave the factory, but after running for a period of time or external damage, water trees and electrical trees are generated and grow. At the same time, with the production of local discharge signals, the insulation is completely deteriorated and even broken down. It is of great significance to investigate the degradation mechanism of cable insulation in order to evaluate the insulation state inside the cables. Before studying the diagnostic method of cable insulation, it is important to probe into the process of cable insulation degradation first.

### 2.1. Degradation Induced by Heating

Thermal-oxidative aging refers to the phenomenon that, being exposed to heat, the chemical structure of insulating medium changes and the insulating properties decrease. The essence of thermal aging is that insulating materials undergo chemical changes under the effect of heat, so thermal aging is also known as chemical aging. Generally speaking, the rate of chemical reaction grows as the ambient temperature increases. The polymeric organic materials used for insulation may undergo thermal degradation under the long-term effect of heat, principally oxidizing reaction. Such kind of reaction is also called autoxidation radical chain reaction. For example, the oxidizing reaction of polyethylene just starts from the disengagement of H from the C-H bond. Thermal aging can degrade the electrical and mechanical properties of insulating materials simultaneously and shorten their insulation life. However, the most evident manifestation is the changes of mechanical properties, such as elongation and tensile strength of materials. In recent years, many scholars have carried out research on the partial discharge characteristics of insulating medium under thermal-oxidative aging and yielded fruitful results [12]. Zhou et al. examined the influence of thermal-oxidative aging time on the electrical tree initiation characteristics of silicone rubber and concluded that the damage of silicone rubber crosslink network at 90°C was an important driver for the sharp decline of the treeing voltage of silicone rubber and changes of electrical trees [13]. Wang et al. investigated the effect of temperature on the discharge characteristics of insulating cardboards with different aging degrees on the dielectric surface and concluded that the higher the degree of aging of cardboard sample is, the more obviously affected it is by temperature. The higher the degree of aging of the cardboard sample is at the high temperature, the more seriously its insulating properties are damaged [14].

### 2.2. Degradation Induced by Chemical Factors

The ambient gases in coal mines have complex composition. Some coal mines, in particular, have corrosive gases such as hydrogen sulfide. Therefore, if sulfide penetrates into cables and insulating sheaths and reacts with copper conductors, compounds such as copper sulfide and copper oxide may be produced. This degradation forms gradually and expands to the sheath of cable, even in the absence of electric field. Under the effect of electric field, the degradation process will be promoted. Due to the high conductivity of chemical trees property, the breakdown voltage of the cable insulation significantly decreases. In addition, the insulating materials of cables are also affected by chemicals, such as lubricating oil and emulsion that drips from underground equipment. The specific effect mode varies with the type of chemicals. Once they permeate the insulating materials of cables, damage such as swelling, lower mechanical strength, and variation in solubility will occur, which weaken cable insulation resistance, harden cables, and lower the breakdown voltage of cables.

### 2.3. Degradation Induced by Water

Water degradation is a form of degradation triggered by water in the coexistence of water and electric field. Water degradation can happen even in a fairly low electric field. In a humid environment in underground coal mines, moisture tends to spread to the irregular areas in the insulation layer of cables and accumulates. Under the long-term effect of electric field, water and some of the media will have chemical reaction and electrochemical reaction. After the decomposition of substances, cavities will be formed. Water fills in the cavities continuously and forms water trees. No discharge can be observed in the expansion areas of water trees. The optical observation of water trees is blurred and there are no branches. It is composed of tiny water droplets and water silk connecting them [15, 16]. After a cable is used for a period of time, the insulation layer will age, mainly because the discharge inside the insulation produces fine crack and forms tiny and hollow channels. On the wall of the channels, there are traces of carbon granules produced by electric discharge, which are few and distinct, just like branches in winter. Under the sustained effect of electric field, the dendritic microchannels run through the whole insulation along the direction of electric field. It is named electric tree, for its shape resembles a dry branch. The channel of electrical tree is hollow, with a diameter of about 10 um. In a transparent solid, its shape, length, and clear outline can be observed under a microscope [17, 18]. Water trees are at high electric field intensity. With the passage of time, they will finally turn into electric trees. Both electric trees and water trees start in the insulation where the electric field is concentrated, that is, where the insulating medium is nonuniform. Under the action of electric field intensity, the local dendritic damage formed in a given area in the insulating material will probably lead to reduced insulation level of the entire cable.

### 2.4. Degradation Induced by Other Factors

If there are gaps or other defects between insulators in the manufacturing process of cables, partial discharge will occur in the gaps between insulators when the cable works, and repeated discharge may gradually corrode the insulators and further reduce the breakdown voltage of the cable [19]. Mechanical damage and deformation are also factors contributing to cable degradation. Due to external damage, the cable can undergo thermal expansion in a short period of time. Together with other factors, the insulating properties of cables will be impaired [20]. Apart from normal operating voltage, there is also unexpected voltage, on-off voltage in case of power supply accidents, switching surge, and lightning surge voltages. These abnormal voltages initiate cable degradation [21]. The structural defects of cable terminals and connectors also give rise to cable degradation. The terminals are not wounded with straps with a cabling degradation cover. Salt and ash fouling will result in leakage and discharge on the surface, and even surface carbonization, and lead to the so-called cabling degradation [22].

## 3. The Principle of Online Monitoring of Insulation of Mine Cables Based on Decision Tree

The 6/10 kV power supply system of underground coal mines has a single-power dendritic structure. The lines in the system are complex and changeable, with different load operation cycles. When a cable has insulation degradation, the zero-sequence voltage and the current of the feed line of the bus in the system show different laws. For this reason, all kinds of zero-sequence parameters of the power supply system of coal mines can be adopted as a basis for subsequent diagnosis of insulation states of cables.

### 3.1. Analysis of Zero-Sequence Parameters of the High-Voltage Power Supply System of Coal Mines

The cable insulation is eroded by moisture, manifested as the increased distributed capacitance in the circuit parameters of cable. When the insulation of a cable fails, it is manifested as the decreased insulation resistance in the circuit parameters of cable, namely, increased insulation conductance. Therefore, in a circuit model, the degradation of cable insulation in any form can be equivalent to connecting large impedance in parallel near the insulation resistance of a certain phase of the cable. As shown in Figure 1, assume that line *L* − *j* had insulation deterioration in a certain phase; in the zero-nematic network, it can be equivalent to adding voltage sources *U*_0_, *I*_1_, *I*_2_,…, *I*_*j*_,… which have the same zero-sequence voltage size and polarity. *I*_*n*_ represents the zero-sequence current of all cable lines, *X*_*L*_ represents the reactance of the arc coil *L*, the insulation value of the cable line is the total insulation guide of the three phases of the cable, and the cable's insulation impedance value is much larger than the line resistance, that is, *Z*_*n*_=1/*Y*_*n*_ ≫ *Z*_*Ln*_ so the effect of line resistance is negligible. In addition, the reactance of the arc coil is much larger than the zero-sequence impedance of the transformer; i.e., the zero-sequence impedance of the transformer is negligible. For a circuit with symmetric insulation, the relationship between its zero-sequence voltage and zero-sequence current satisfies the following equation:

(1) $$\begin{array}{c} I_{i}=jwC_{i}\cdot U_{0}+G_{i}\cdot U_{0}. \end{array}$$

It is simple to analyze the single-phase insulation degradation of cables. Suppose that the a-phase insulation of the cable *L*-*j* degrades. As shown in Figure 2, for the a-phase with degraded insulation, its insulation admittance is equivalent to adding a parallel conductance to the original insulation admittance. *Y*_*a*_, *Y*_*b*_, and *Y*_*c*_ represent original three-phase insulation admittance, respectively, are defined as the reciprocal of the impedance according to Power Electronics, and are used to describe the difficulty level of the alternating current passing the circuit or system. Admission is a vector, consisting of scalar conductivity and electrical susceptance. In the figure *G*_*a*_, *G*_*b*_, and *G*_*c*_ are the three-phase insulation conductance of cable *L*-*j* to ground, *C*_*a*_, *C*_*b*_, and *C*_*c*_ are the three-phase distributed capacitance of cable *L*-*j* to ground, *U*_*a*_, *U*_*b*_, and *U*_*c*_ are the three-phase power phase voltage of the system, *U*_0_ is the zero-sequence voltage of the neutral point of transformer, and the zero-sequence voltage of each point in the system is equal to the zero-sequence voltage of the neutral point of transformer. *G*_*xj*_ is the equivalent conductance of the a-phase with degraded insulation. Except the equivalent conductance of degraded phase, the insulation values of the three phases of the cable are equal, i.e., *G*_*a*_=*G*_*b*_=*G*_*c*_, *C*_*a*_=*C*_*b*_=*C*_*c*_

According to Kirchhoff's circuit law, the zero-sequence current of cable *L*-*j* is

(2) $$\begin{array}{c} I_{j}=\left(U_{a}+U_{0}\right)\left(Y_{a}+G_{xj}\right)+\left(U_{b}+U_{0}\right)Y_{b}+\left(U_{c}+U_{0}\right)Y_{c}, \end{array}$$

where *Y*_*a*_=*G*_*a*_+*jwC*_*a*_, *Y*_*b*_=*G*_*b*_+*jwC*_*b*_, *Y*_*c*_=*G*_*c*_+*jwC*_*c*_, and *Y*_*a*_=*Y*_*b*_=*Y*_*c*_. Even if the cable in the system is no longer completely symmetric in three phases, the voltage sum of the three phases of the system power supply is always 0, that is, *U*_*a*_+*U*_*b*_+*U*_*c*_=0. To substitute it into equation (2), we have

(3) $$\begin{array}{c} {\dot{I}}_{j}={\dot{U}}_{0}\left(Y_{a}+Y_{b}+Y_{c}\right)+\left({\dot{U}}_{a}+{\dot{U}}_{0}\right)G_{xj}={\dot{U}}_{0}Y_{j}+\left({\dot{U}}_{a}+{\dot{U}}_{0}\right)G_{xj}, \end{array}$$

where *Y*_*j*_=*Y*_*a*_+*Y*_*b*_+*Y*_*c*_ is the admittance of the symmetric insulation part of this cable. Since the cable length is short and the distributed capacitance is small, *Y*_*j*_ is small, and *U*_0_*Y*_*j*_ is negligible; thus we can approximately get the insulation resistance to ground as follows:

(4) $$\begin{array}{c} R_{xj}=\frac{U_{a}+U_{0}}{I_{j}}. \end{array}$$

As can be seen from equation (3), the production of zero-sequence voltage is the result of the joint effect of the phase voltage of the degraded a-phase, the equivalent conductance *G*_*xj*_, and the admittance *Y*_*j*_ of the symmetric part of insulation. According to equation (3), the internal equivalent circuit of zero-sequence voltage at the terminals *a* and *b* in Figure 2 can be simplified as Figure 3. As cable a-phase has deterioration, the equivalent conductance *G*_*xj*_ is parallel connected to the original equivalent circuit, making zero-sequence current and the zero-sequence voltage of the cable change accordingly.

After integrating Figures 1 and 3, we can form a new equivalent circuit, as shown in Figure 4. It can be seen that, due to the deterioration of a-phase of line *L* − *j*, the equivalent conductance *G*_*xj*_ has increased, which is different with the equivalent circuit of other lines.

When the neutral point of the power supply system is not grounded, through Kirchhoff's voltage law, the relationship between the zero-sequence voltage and the phase voltage of the system can be obtained as follows:

(5) $$\begin{array}{c} {\dot{U}}_{0}=-\frac{{\dot{U}}_{a}G_{xj}}{G_{\sum }+G_{xj}+jwC_{\sum }}=-\frac{{\dot{U}}_{a}G_{xj}}{\sqrt{{\left(G_{\sum }+G_{xj}\right)}^{2}+w^{2}C_{\sum }^{2}}}e^{-j\theta }, \end{array}$$

where *θ*=arctan{*wC*_Σ_/(*G*_Σ_+*G*_*xj*_)} and *θ* ∈ (0, 90°). So the phase angle that the zero-sequence voltage ${\dot{U}}_{0}$ lags behind the phase voltage ${\dot{U}}_{a}$ of the insulation degradation phase is within (90° ~ 180°). *G*_Σ_=*G*_1_+*G*_2_+⋯+*G*_*j*_+*G*_*n*_ is the distributed capacitance value of the total symmetric part of the system. When the neutral point of the system is grounded via the arc suppression coil, the relationship between the zero-sequence voltage and the phase voltage of the system is as follows:

(6) $$\begin{array}{c} U_{0}=-\frac{U_{a}G_{xj}}{G_{\Sigma }+G_{xj}+j\left(wC_{\Sigma }-1/wL\right)}=-\frac{U_{a}G_{xj}}{\sqrt{{\left(G_{\Sigma }+G_{xj}\right)}^{2}+{\left(wC_{\Sigma }-1/wL\right)}^{2}}}e^{-j\theta }, \end{array}$$

where *θ*=arctan{*w*(*C*_Σ_ − 1/*wL*)/(*G*_Σ_+*G*_*xj*_)}.

Overcompensation is a frequently used compensation mode in the power grids of coal mines, that is, *wC*_Σ_ < 1/*wL*, so *θ*=(−90°, 0). The phase angle at which the zero-sequence voltage *U*_0_ stays ahead of the phase voltage ${\dot{U}}_{a}$ of the insulation degradation phase is within 90°∼180°.

When the insulation of a given phase of the high-voltage cable degrades, the system parameters will lose balance, making the system generate zero-sequence voltage. To make the system regain balance, other cables with normal insulation will generate zero-sequence current accordingly [23, 24]. As shown in Figure 5, the zero-sequence voltage *U*_0_ is taken as the reference phasor, and the angle *φ*(*φ*=180° − *θ*) between the phase voltage and the zero-sequence voltage *U*_*a*_ changes dynamically. According to equations (4) and (5), the degree of change is related to the total insulation parameter value of the system and the grounding mode of the neutral point.

*U*_*a*  *d*_=*U*_*a*_+*U*_0_ is the voltage to ground of a-phase, and *I*_1_, *I*_*n*_ are zero-sequence currents of cables with normal insulation, whose angle with the zero-sequence voltage of the system is proximate to 90°.

${\dot{I}}_{j}={\dot{I}}_{j0}+{\dot{I}}_{xj}$ is the zero-sequence current of the cable with degraded insulation. It is formed by superimposing the zero-sequence current ${\dot{I}}_{j0}$ generated by the three-phase symmetric admittance of this cable and the current formed by the equivalent conductance *G*_*xj*_ of the insulation degradation phase. Thus, it can be concluded that there is a great difference between the phase of the zero-sequence current of the cable with degraded asymmetric insulation and that of the cable with symmetric insulation.

To sum up, the relation vector between the zero-sequence voltage and zero-sequence current of the cable with symmetric insulation in the power supply system is different from the relation vector between the zero-sequence voltage and zero-sequence current of the cable with single-phase insulation degradation. The grounding mode of the neutral point of the power supply system has an impact on the zero-sequence voltage of the system but does not affect the relation vector between the zero-sequence component of the cable line itself and the insulation parameters. The degradation types of cable insulation include not only single degradation, but also two degradations and three symmetric degradations, but the probability of three completely symmetric degradations of insulation is almost zero [25].

### 3.2. Decision Tree for the Degradation of Cable Insulation Evaluation

The total insulation resistance of cables in underground coal mines can be regarded as the parallel connection of three insulation resistances and denoted as *r*∑. The insulation resistance of underground cables can be classified into three types: good (to be used normally), dangerous (to be monitored emphatically), and highly dangerous (to be replaced). The evaluation criteria are shown in Table 1.

The insulation state of the cables in coal mines can be divided into two types: symmetric insulation and asymmetric insulation. Symmetric insulation can be further divided into normal insulation and degraded symmetric insulation, while asymmetric insulation can be further divided into single-phase insulation degradation and two-phase insulation degradation [26].

#### 3.2.1. Decision Subtree for the Symmetry of Cable Insulation

Suppose that the insulation of the cable is symmetric and satisfies equation (1); then the following equation can be established:

(7) $$\begin{array}{c} i_{i}=C_{i}\frac{du_{o}}{dt}+G_{i}\cdot u_{o}. \end{array}$$

The zero-sequence current and zero-sequence voltage in equation (6) are sampled synchronously, and multiple points are collected on an ongoing basis. The midpoint method is used to find the derivative of zero-sequence current. The equation is as follows:

(8) $$\begin{array}{c} \frac{du_{o}}{dt}\left(k\right)=\frac{u_{o}\left(k+1\right)-u_{o}\left(k-1\right)}{2\Delta t}, \end{array}$$

where Δ*t* is the step size. An appropriate step size is selected and then *k* sets of data are selected at equal intervals to build the following overdetermined equation set:

(9) $$\begin{array}{c} \left[\begin{array}{cc} \frac{du_{0}}{dt}\left(1\right) & u_{0}\left(1\right)\\ \frac{du_{0}}{dt}\left(2\right) & u_{0}\left(2\right)\\ \vdots & \vdots \\ \frac{du_{0}}{dt}\left(k\right) & u_{0}\left(k\right) \end{array}\right]\cdot \left[\begin{array}{c} C_{1}\;\;\;\;\;\;\;\;\;\;C_{2}\;\;\;\;\;\;\;\;\;\;\cdots \;\;\;\;\;\;\;\;\;\;C_{n}\\ G_{1}\;\;\;\;\;\;\;\;\;\;G_{2}\;\;\;\;\;\;\;\;\;\cdots \;\;\;\;\;\;\;\;\;\;G_{n} \end{array}\right]=\left[\begin{array}{c} \;\;i_{1}\left(1\right)\;\;\;\;\;\;\;\;\;\;\;i_{2}\left(1\right)\;\;\;\;\;\;\;\;\;\;\cdots \;\;\;\;\;\;\;\;\;\;i_{n}\left(1\right)\\ \;i_{1}\left(2\right)\;\;\;\;\;\;\;\;\;\;i_{2}\left(2\right)\;\;\;\;\;\;\;\;\;\cdots \;\;\;\;\;\;\;\;\;i_{n}\left(2\right)\\ \;\;\;\;\;\;\;\;\vdots \;\;\;\;\;\;\;\;\;\;\;\;\;\;\;\;\;\;\;\;\;\;\;\;\;\;\;\vdots \;\;\;\;\;\;\;\;\;\;\;\;\;\;\;\;\;\ddots \;\;\;\;\;\;\;\;\;\;\;\;\;\;\;\;\vdots \\ i_{1}\left(k\right)\;\;\;\;\;\;\;\;\;\;i_{2}\left(k\right)\;\;\;\;\;\;\;\;\cdots \;\;\;\;\;\;\;\;i_{n}\left(k\right) \end{array}\right]. \end{array}$$

*n* represents the serial number of the cable line, and *k* represents the number of sets of data selected at equal intervals.

#### 3.2.2. Decision Subtree for the Diagnosis of Single-Phase Insulation Degradation

The relationship between the zero-sequence components of the cable with single-phase insulation degradation meets equation (3). The following differential equation is established according to equation (3):

(10) $$\begin{array}{c} i_{j}=C_{j}\frac{du_{o}}{dt}+G_{j}\cdot u_{o}+G_{xj}\cdot u_{ad}. \end{array}$$

The insulation parameter of the cable can be solved by collecting *k* sets of data synchronously at equal intervals:

(11) $$\begin{array}{c} {\left[C_{J}\;\;\;\;\;\;\;\;\;G_{j}\;\;\;\;\;\;\;\;\;\;\;G_{xj}\right]}^{T}={\left(A^{T}A\right)}^{-1}\cdot A^{T}\cdot b. \end{array}$$

where *C*_*j*_, *G*_*j*_ are the conductance and capacitance value of single-phase insulation deterioration lines.

(12) $$\begin{array}{c} A=\left[\begin{array}{ccc} \frac{du_{0}}{dt}\left(1\right) & u_{0}\left(1\right) & u_{a\;d}\left(1\right)\\ \frac{du_{0}}{dt}\left(2\right) & u_{0}\left(2\right) & u_{ad}\left(2\right)\\ \vdots & \vdots & \vdots \\ \frac{du_{0}}{dt}\left(k\right) & u_{0}\left(k\right) & u_{ad}\left(k\right) \end{array}\right],\\ b=\left[\begin{array}{c} i_{j}\left(1\right)\\ i_{j}\left(2\right)\\ \vdots \\ i_{j}\left(k\right) \end{array}\right],\\ k>3. \end{array}$$

The total insulation conductance of the cable *L*-j is the sum of all conductance values.

(13) $$\begin{array}{c} G_{J\sum }=G_{J}+G_{xj}. \end{array}$$

#### 3.2.3. Diagnosis Decision of Two-Phase Insulation Degradation

When a cable has two insulation degradations, it can be expressed as follows in the form of a differential equation:

(14) $$\begin{array}{c} i_{j}=C_{j}\frac{du_{o}}{dt}+G_{j}\cdot u_{o}+G_{xja}\cdot u_{ad}+G_{xjb}\cdot u_{ad}. \end{array}$$

Through matrix calculation, the insulation parameter of the cable is

(15) $$\begin{array}{c} {\left[C_{J}G_{j}G_{xja}G_{xjb}\right]}^{T}={\left(A^{T}\cdot A\right)}^{-1}\cdot A^{T}\cdot b \end{array}$$

where $A=\left[\begin{array}{c} du_{0}/dt\left(1\right)u_{0}\left(1\right)u_{ad}\left(1\right)u_{bd}\left(1\right)\\ du_{0}/dt\left(2\right)u_{0}\left(2\right)u_{ad}\left(2\right)u_{bd}\left(2\right)\\ \vdots \vdots \vdots \vdots \\ du_{0}/dt\left(k\right)u_{0}\left(k\right)u_{ad}\left(k\right)u_{bd}\left(k\right) \end{array}\right]$, $b=\left[\begin{array}{c} i_{j}\left(1\right)\\ i_{j}\left(2\right)\\ \;\;\;\;\;\;\;\vdots \\ i_{j}\left(k\right) \end{array}\right]$, *k* > 4.

At this point, the insulation conductance of phases *a* and *b* and the total conductance of the line are

(16) $$\begin{array}{c} \left\{\begin{array}{c} G_{ja}\;\;\;\;\;=\frac{G_{j}}{3}+G_{Xja},\\ G_{jb}\;\;\;\;\;=\frac{G_{j}}{3}+G_{Xjb},\\ G_{j\sum }=G_{j}+G_{Xja}+G_{Xjb}. \end{array}\right. \end{array}$$

## 4. Verification of the Degradation Judgment Method Based on Decision Tree through Simulation

To verify the effectiveness of the degradation judgment method based on decision tree, the author sets up a simulation experiment for the purpose of simulation calculation and verification. The power grid of underground coal mines is simulated, and Matlab simulation software is used to set up a single-power dendritic power supply system. 5 cables are selected to form a single-power dendritic power supply system, and a simulation model to diagnose the insulation state of cables is built. The parameters of cable lines in the simulation model are shown in Table 2 below.

Suppose that the zero-sequence voltage, phase voltage, and the zero-sequence current of all lines in the simulated power supply system are collected synchronously. Since the grounding mode of the neutral point of the system does not influence the judgment method of the decision tree, a system where the neutral point is not grounded is taken as a simulation model to verify the effectiveness of the decision method. Table 2 is the parameters of all cable lines, including model, length, and load. The parameters of each line with normal insulation in the simulation model are shown in Table 3.

None of the loads in the coal mine power grid are grounded, and the relationship between the zero-sequence component and insulation parameters of each cable branch is not affected by the loads, so the loads can be simplified during the simulation. The active load powers of the lines are 315 kW, 250 kW, 560 kW, 1250 kW, and 630 kW. The sampling rate is set to 100 kS/s and the step size is set to 1 us.

Run the simulation model, and the zero-sequence voltage waveform of the simulation system is shown in Figure 6. All cable lines in simulation settings (Table 2) have symmetric and good insulation within 0–0.01 s and Line L2 has c-phase insulation degradation at 0.01 s, the c-phase insulation conductance decreases to 2 × 10^−6^ S, and the insulation of the other two phases has not changed. Line L4 has insulation degradation in phases *b* and *c* at 0.05 s, the conductance of both phases *b* and *c* drops to 3 × 10^−7^ S, and the insulation of a-phase does not deteriorate and the simulation duration is 0.15 s.

The simulation model is run, and the zero-sequence current waveform of each simulated cable is shown in Figure 7. Within the time frame of 0–0.01 s, the three-phase symmetric insulation, zero-sequence voltage, and zero-sequence current of all lines in the system are 0. At 0.01 s, the c-phase insulation of the line L2 degrades, zero-sequence voltage appears in the system, and zero-sequence current is generated in each line. At 0.05 s, the insulation of phases *b* and *c* in line L4 degrades, and the zero-sequence voltage of the system and the zero-sequence current of each line change. In addition, it can be seen that there exists a DC component in the zero-sequence voltage, which can be ascribed to the charge and discharge of the distributed capacitance of the lines. The changes of zero-sequence voltage and zero-sequence current in Figures 6 and 7 prove the correctness of the simulation model.

## 5. Analysis of Online Monitoring Solutions for Cable Insulation

Currently, the mainstream online monitoring methods for cable insulation in China include DC superposition method, DC component method, AC superposition method, partial discharge method, and dielectric loss method [27].

The DC superposition method is to apply a 50 V low-voltage DC to the normal running cable at the grounding site of the neutral point of the voltage transformer, to measure the weak DC current passing through the insulation layer of cable or its insulation resistance, so as to judge the aging degree of the cable. The shortcoming of this method is that when the DC current passes through the voltage transformer for a long time, it will make the magnetic circuit of the transformer saturated and generate zero-sequence voltage, resulting in misoperation of the substation relay [28]. The DC component method is to judge the aging degree of cables by measuring the DC leakage current produced by the rectification of water trees of cables. It is not suitable for newly laid cables and dry cross-linked cables without water trees [29]. The partial discharge method is to apply a relatively high voltage to the main insulation of the cable to measure the partial discharge at the defective part of cable under the joint effect of electric field, heat, and machinery, etc. and judge the damage degree of the main insulation based on the amount of discharge. The defect of the partial discharge method is that, due to the complexity of discharge signal, it is impossible to realize real-time monitoring [30]. The AC superposition method is to superimpose an AC voltage of 2 times of power frequency plus 1 Hz on the shielding layer of cable in operation, to detect 1 Hz current signal with AC features, so as to judge the aging of the cable. For networks whose neutral points are directly grounded, neither the DC superposition method nor the AC superposition method applies [31]. The dielectric loss tangent measurement method can monitor the overall defects of the cable but cannot reflect the local degradation of insulation, so this method shall be integrated with other methods. The dielectric loss method calculates the dielectric loss factor (tan*δ*) of cable insulation by collecting the core voltage and current signal to ground of the cable, so as to reflect the defects of the cable, such as damp, joint aging, or water tree degradation [32]. Due to the need to input low-frequency signals and complex operation, the dielectric loss method is suitable for the temporary test of cable insulation.

Due to the special environment in underground coal mines, so far, underground power grids generally apply the insulation monitoring method based on zero-sequence voltage and the leakage protection method based on power direction. Both of them have certain limitations. The insulation monitoring based on zero-sequence voltage cannot show the change after the three-phase symmetric insulation of the power grid declines. The shortcoming of the leakage protection based on power direction is that a trip signal will not be sent unless electricity leaks from the cable. It is impossible to predict the insulation level of power grid accurately before a ground fault occurs. Compared with the ground power transmission and distribution system, high-voltage cables under the shaft are characterized by short length of cable, nonunified grounding mode of the shielding layer of cable, and many types of cables, etc. Since the current online monitoring methods of insulation in the power grids of underground coal mines have different defects, it is important to explore new online monitoring methods of insulation.

## 6. Wide-Area Synchronous Measurement and Monitoring System for Cable Insulation

In this paper, we intend to explore a cable insulation monitoring method based on wide-area synchronous measurement. The proposed method can only acquire three voltages, zero-sequence voltage, and zero-sequence current at one end of a cable synchronously and directly calculate its insulation resistance.

### 6.1. Design of Timing System

The automation device of power system has an in-built real-time clock, or there is a GPS-dominated timing device inside the station. However, it is hard to avoid the inherent errors. With the increase of operation time, the cumulative error is getting bigger and bigger, making it difficult to describe the chronological order accurately and posing certain difficulties to the analysis of power grid faults. How to synchronize the real-time time with the clock and unify the time of the whole network is a goal that has long been sought after by the power system. GPS (Global Positioning System) is the most widely used and accurate time release system in the world. However, the United States does not assume responsibility for its civilian users and does not guarantee the accuracy and reliability of GPS clock [33]. In the case of the loss of lock of the satellite or experimental jump of satellite clock, the error of GPS clock can reach one hundred ms [34]. The Compass Navigation Satellite System (CNSS) is a satellite navigation system independently developed by China. CNSS system can offer all-weather, fast, and high-precision timing functions for users in the service area and has such advantages as being safe, stable, and reliable, which is beyond comparison by GPS system. Therefore, the wide-area synchronous measurement system adopts the CNSS system from China for timing and realizes high-precision timing, with a timing precision of up to 60 ns–5 ns.

The high precision of CNSS timing can ensure that the relative error between the time signals and UTC will not exceed 20–100 ns and realize real synchronization of the whole network, as well as the synchronization management of time and remote monitoring of the whole power network [35]. The principle of CNSS timing is similar to that of GPS timing, except that there are two timing modes: active and passive. One is two-way time lag transmission, and the other is broadcast timing. An active receiver needs an SIM card, and its timing frequency is restricted by the use frequency of the card, so generally speaking, such kind of receiver cannot merely be used as a professional timing device. A passive receiver only demodulates messages, and passive timing receivers are further divided into two-satellite receiver and three-satellite receiver. As a two-satellite passive CNSS receiver cannot assign accurate time unless accurate longitude, latitude, and altitude coordinates are input, it is not convenient for engineering installation and use and cannot meet the demand of dynamic timing, while a three-satellite receiver can achieve high-precision timing as long as accurate altitude is input. Moreover, if there is sustained input of altitude, dynamic timing application can be satisfied. With this in mind, the synchronous measurement system adopts a three-satellite receiver to achieve high-precision timing, that is, to provide reliable clock source, synchronization management of time of the whole network, and remote real-time monitoring and maintenance.

### 6.2. Design of a Wide-Area Synchronous Online Measurement and Monitoring System for Cable Insulation

Consider that the smart grid is an interoperable system [36], which requires a synchronous phasor measurement unit (PMU) with simple structure and clear functions [37, 38]. The wide-area synchronous measurement system is composed of four parts: global positioning system (CNSS), signal collector, measuring unit (PMU monitoring substation), and communication network and control center.

The basic principle of PMU monitoring substation is that the filtered AC signal is quantized by the A/D converter, and the microprocessor calculates the phasor based on the preset algorithm. According to the form specified in IEEE Std 1344–1995, positive-sequence phasor, time stamp, etc. are assembled into messages and transmitted to the host of monitoring center on the ground through the optical network. The monitoring host collects information from all PMU monitoring substations, in order to provide data for the monitoring, protection, and control of the whole system.

As shown in Figure 8, PMU monitoring substations consist of power circuit, CNSS receiving module, microprocessor, communication module, data acquisition circuit, display, alarm, status indication and management interface, etc. The 127 V AC power supply for mines offers power for each functional module, through the conversion of the power modules AC/DC and DC/DC. The analog signal input of cable insulation parameter is converted to a digital signal through the high-speed AD circuit and assigns time information via the CNSS timing module, which is uploaded by the communication module after being processed by the microprocessor. The substation property has such functions as LCD display, status indication, overlimit alarm, and external management.

The synchronous acquisition of the phase voltage, zero-sequence voltage, and zero-sequence current of each line is achieved by wide-area synchronous measurement technology. The signal collector collects zero-sequence voltage through the secondary winding of the three-phase five-column voltage transformer. The zero-sequence current is collected by the signal collector through the zero-sequence current transformer in the high-explosive switch of the cable feeder. The signal collector communicates with the PMU monitoring substation in real time to realize the acquisition and uploading of signals. The measured data are uploaded to the monitoring host through the high-speed optical network. After the monitoring host collects the zero-sequence current of various cable feeders, as well as the zero-sequence voltage and phase voltage of the system, it judges the insulation state of cables via the online real-time monitoring software for cable insulation.

### 6.3. Judgment of Cable Insulation Level

To overcome the limitation that the voltage and current at any part of the cable cannot be measured accurately without prejudice to the integrity of cable, the terminal voltage and terminal current of the cable are selected as measurements for analysis and calculation, in order to get the original parameters of the whole cable and judge the insulation state of the cable.

As shown in Figure 9, the ground monitoring host communicates with PMU monitoring substation in real time through the high-speed optical network, captures the running state of various underground cables, dispatches power supply rationally, and ensures that the overhauled cable runs without any load. The dielectric loss tangent (tan*δ*) of a cable can be calculated by collecting the voltage to ground and line current of this cable synchronously at high speed. At the same time, the insulation resistance of the cable can be calculated, which can truly demonstrate the insulation level of the cable.

The specific process is as follows:

1. The zero-sequence voltage and phase voltage of the system and the zero-sequence current of all lines are time-stamped with a CNSS synchronous timing module, and the insulation parameters of all lines are calculated through equation (8). It should be noted that when there is a subordinate substation in a cable, the zero-sequence current in equation (8) shall be equal to the zero-sequence current of this cable minus the zero-sequence current of all feeders in the subordinate substation.
2. If both the insulation conductance and distributed capacitance in the calculation results are positive, the insulation state of the cable can be judged according to the criteria in Table 1. If there is a negative value for insulation conductance or distributed capacitance of a given cable in the calculation results, the insulation of this cable is identified to be degraded asymmetrically.
3. For cables with asymmetric insulation, if the zero-sequence Δ*I*_*j*_ is in the same phase with the voltage to ground of a given phase of the system, it is judged that the insulation of this phase degrades. If the phase of the zero-sequence variation Δ*I*_*j*_ falls between the phases of the voltages to ground of two phases, it is judged that both phases have degraded asymmetric insulation.
4. For cables with single-phase insulation degradation, the control center calculates the insulation parameter of the cable with equations (9) and (10). For cables with two-phase insulation degradation, it calculates the insulation parameter of the cable with equations (13) and (14).

After that, based on the calculation results, the insulation states of lines are classified, and the parameter values and insulation state are displayed by class on the LCD. If there is any cable “to be replaced immediately,” an alarm will be given.

## 7. Application and Effect of the Insulation Monitoring Technology for High-Voltage Cables in Coal Mines Based on Decision Tree

In this paper, the criteria or insulation status diagnosis and the detailed decision tree to realize the classification of insulation were provided. Considering the influence of the load three-phase imbalance on the decision tree method, this paper pointed out the difference between the load neutral-point ungrounding and neutral-point grounding when establishing the insulating tree and determined the modification method when applying the decision tree method to the load grounding system. The feasibility of the method was verified by simulation experiments. The application of the insulation monitoring technology of high-voltage cables in underground coal mines based on decision tree indicates that the phase voltage and zero-sequence voltage of the system and the zero-sequence current of all lines are all easy to collect and suitable for the calculation of the insulation parameters of cables. When this method is adopted to diagnose insulation online, the change in the zero-sequence current of cable can be monitored ceaselessly, which can help improve the accuracy of decision-making.

The insulation monitoring technology of high-voltage cables in underground coal mines based on decision tree has been popularized and applied in substations of multiple coal mine enterprises in China, such as China Shenhua Energy Company Limited Shendong Coal Branch, Erdos Haohua Hongqingliang Mining Co., Ltd., Shanxi Hoerxinhe Coal Industry Co. Ltd., etc., which solves the difficulty in real-time monitoring of the degradation of cable insulation in coal mines. Ever since the insulation monitoring devices of high-voltage cables in underground coal mines based on decision tree were put into use, they can achieve the full coverage of the monitoring of insulation degradation of high-voltage cables in underground coal mines, timely and accurately monitor the changes of cable insulation, and give alerts promptly. The development and application of the system effectively minimize underground power outages induced by the degradation of cable insulation and avoid secondary disasters under the mines caused by power outage. It is possible to identify hidden cable degradation in time, troubleshoot cable degradation accurately, and improve the ability to guarantee the safety of power supply in underground coal mines.

## Figures and Tables

**Figure 1:** Simplified diagram of zero-sequence network.

**Figure 2:** Equivalent arithmetic circuit diagram of the cable with degraded insulation.

**Figure 3:** Internal equivalent circuit of zero-sequence voltage in the cable with single-phase insulation degradation.

**Figure 4:** Zero-sequence equivalent circuit of the cable with single-phase insulation degradation.

**Figure 5:** The current relation vector of zero-sequence network.

**Figure 6:** Zero-sequence voltage waveform.

**Figure 7:** Zero-sequence current waveform of the lines.

**Figure 8:** Functional structure of the PMU monitoring substation.

**Figure 9:** Block diagram of the insulation monitoring structure of the high-voltage cables in coal mines based on decision tree.

**Table 1:** The evaluation criteria of insulation states of cables.

Indicator	Measurement (MΩ)	Evaluation	Decision	Class
Insulation resistance of the cable tested	*r*∑ ＞ 10	Good	To be used	*W*_1_
	1 ＜ *r*∑ ≤ 10	Dangerous	To be monitored emphatically	*W*_2_
	*r*∑ ≤ 1	Highly dangerous	To be replaced	*W*_3_

**Table 2:** Parameters of cable lines in the simulation model.

Line	Number of cores × nominal cross section (mm × mm^2^)	DC resistance at 20°C (*ω*/km)	Insulation thickness (mm)	Length of line (km)	Active load power (kw)
L1	3 × 120	0.153	4.5	2.5	315
L2	3 × 185	0.099	4.5	0.57	250
L3	3 × 240	0.075	4.5	1.9	560
L4	3 × 150	0.124	4.5	0.3	1250
L5	3 × 95	0.193	4.5	1.3	630

**Table 3:** Insulation parameters of the lines in simulation model.

Line	L1	L2	L3	L4	L5
Insulation conductance of each phase (∗10^−8^S)	2.5	0.57	1.90	0.3	1.3
Distributed capacitance of each phase (uF)	0.2718	0.0961	0.3204	0.0357	0.1300

## Data Availability

No data were used to support this study.
